# Effectiveness of Repetitive Facilitative Exercise Combined with Electrical Stimulation Therapy to Improve Very Severe Paretic Upper Limbs in with Stroke Patients: A Randomized Controlled Trial

**DOI:** 10.1155/2022/4847363

**Published:** 2022-04-27

**Authors:** Hitoshi Ohnishi, Hiroyuki Miyasaka, Naoki Shindo, Kazuki Ito, Shiori Tsuji, Shigeru Sonoda

**Affiliations:** ^1^Fujita Health University Nanakuri Memorial Hospital, 424-1, Oodori-cho, Tsu, Mie 514-1295, Japan; ^2^Department of Rehabilitation Medicine II, School of Medicine, Fujita Health University, 424-1, Oodori-cho, Tsu, Mie 514-1295, Japan

## Abstract

**Background:**

The difference in the effects of combined therapy with repetitive facilitative exercise (RFE) and neuromuscular electrical stimulation (NMES) on stroke upper limb paralysis was only reported by a pilot study; it has not been investigated in many patients.

**Objective:**

We investigated the effect of combined therapy with RFE and NMES on stroke patients with severe upper paresis.

**Methods:**

This study included 99 of the very severe paresis stroke patients with scores of zero or 1a in the Finger-Function test of the Stroke Impairment Assessment Set (SIAS). We randomly divided the patients into four groups, namely, NMES, RFE, RFE under NMES, and conventional training (CT) groups. A total of 20 min of group-specific training in addition to 40 min of conventional exercise per day, seven times a week for 4 weeks after admission, was performed. The upper extremity items of the Fugl-Meyer Assessment (FMA) were evaluated before and after the training period.

**Results:**

The total score gains of the FMA, FMA wrist item, and FMA finger item were significantly larger in the RFE under NMES group than those in the CT group (*p* < 0.05).

**Conclusion:**

The combination of voluntary movement and electrical stimulation may promote the activation of paralyzed muscles and improve distal function for very severe paralyzed upper limbs.

## 1. Introduction

Repetitive facilitative exercise (RFE) is a training method for the paralyzed limbs developed by Kawahira et al. RFE facilitates increased excitation of the corresponding injured descending motor tracts using stretch or skin-muscle reflexes elicited immediately before or simultaneously with patient effort to move his or her hemiplegic upper or lower limb [1]. Shimodozono et al. reported that RFE significantly improved the upper limb total Fugl-Meyer Assessment (FMA) and Action Research Arm Test (ARAT) scores as compared to the conventional therapy in patients with subacute stroke [2]. In recent years, the combination of several rehabilitation techniques is reportedly more effective for the functional improvement of paralyzed upper extremities than rehabilitation using only one technique [3, 4]. Moreover, electrical stimulation combined with an upper limb rehabilitation technique such as mirror therapy [5] and robot-assisted therapy [6] further improved recovery from motor paralysis in patients with stroke.

Shimodozono et al. reported the effects of training combined with RFE and NMES (RFE under NMES) in 27 subacute stroke patients with severe upper limb paralysis [7]. The patients were randomly allocated to RFE under the NMES, RFE, and control groups and received each treatment for 40 min per day, five times per week for 4 weeks. The FMA upper limb total score improvement in the RFE under the NMES group was significantly larger than that in the control group. However, this study included few patients, and the combination results were not directly compared to the group in which only NMES was administered.

To address insufficiencies, the present study compared motor paralysis improvements in the upper extremities among four groups (RFE under NMES, RFE only, NMES only, and control groups) with at least 20 patients in each group.

## 2. Materials and Methods

### 2.1. Subjects

The subjects were 1,830 stroke patients admitted to the Fujita Health University Nanakuri Memorial Hospital between August 2011 and July 2015. The inclusion criteria were (1) first-ever stroke and (2) Finger-Function items score in the Stroke Impairment Assessment Set (SIAS) [8, 9] on admission of 0 or 1a. The exclusion criteria were (1) serious comorbidity interfering with training (Liu's comorbidity index [10] of 4 or higher); (2) comprehension item score of the Functional Independence Measure (FIM) < 3 or expression item score of the FIM < 2; (3) using a pacemaker; or (4) inability to maintain a sitting position. After applying these criteria, the present study finally included 101 subjects. The study was approved by the ethical committee of our university (ethical approval number 91). All participants provided written informed consent, and all procedures complied with the principles of the Declaration of Helsinki.

### 2.2. Study Design

This study was a single-center, single-blind randomized controlled trial. Moreover, the evaluator was the occupational therapist. The patients were allocated into one of four groups (NMES, RFE, RFE under NMES, and conventional therapy [CT]) using a computer-generated random number table.

The patients in all groups received 1 hour of exercise per day, seven times per week for 4 weeks. Ten minutes per hour were used for each allocated training method to the proximal part of the affected upper extremity, 10 min to the distal part, and the remaining 40 min were assigned to conventional exercise. The exercise contents in the CT group were 60 min of conventional therapy.

### 2.3. Interventions

#### 2.3.1. NMES Group

The normal mode of the PAS system (OG Giken, Okayama, Japan) was used to induce NMES. The NMES frequency was 50 Hz, and pulse width was 50 *μ*sec. Stimulation continued for 5 sec in maximum allowable intensity level with duty ratio of 1 : 1.

Electrodes were attached to the anterior and middle fibers of the deltoid muscle to stimulate the proximal region and extensor digitorum and extensor carpi radialis to stimulate the distal region. Patients did not intend to move their upper limb during stimulation application.

#### 2.3.2. RFE Group

The tasks for the proximal (shoulder joint flexion and elbow joint flexion-extension) and distal (wrist joint dorsiflexion, extension and opposition of the thumb, and extension of each finger) regions were repeated 100 times or more per 10 min.

#### 2.3.3. RFE under NMES Group

Although the NMES parameters and stimulation regions were the same as those in the NMES group, the electrical stimulation intensity was set to a submotor threshold level without joint movement. NMES was continuously delivered during RFE training.

RFE was performed as described in the RFE group.

#### 2.3.4. CT Group

The CT consisted of passive joint movement, repetitive tasks using objects, or activities of daily living (ADL) exercises. RFE and NMES were prohibited for use.

### 2.4. Determination Criteria of the Target Muscle

The target muscles in the NMES, RFE, or RFE under NMES groups were determined according to the following criteria.

Proximal regions:

The anterior and middle fibers of the deltoid muscle were chosen as the target muscles in patients with scapulohumeral joint subluxation or without any voluntary shoulder joint movement. The triceps was selected as the target muscle in patients with any shoulder movement and with exaggerated tonus or weakened triceps brachii muscle.

Distal regions:

The extensor carpi radialis muscles were targeted in patients without any voluntary movement of the wrist extension. The extensor digitorum muscle was used as the target muscle in patients with any movement of the wrist extension and without volitional movement of the finger extension.

### 2.5. Assessment

The SIAS Knee-Mouth and Finger-Function tests, shoulder/elbow, wrist, finger, and upper limb total FMA score, Modified Ashworth Scale (MAS) at the biceps brachii muscle and wrist flexors and the FIM score were evaluated on admission and 4 weeks after admission. The SIAS comprises items examining motor function, muscle tone, sensory function, range of motion, pain, trunk balance, visuospatial perception, aphasia, and function of the unaffected side [8, 9]. The Knee-Mouth and Finger-Function tasks include elevation of the affected upper extremity to the mouth and individual flexion and extension of the five digits, respectively. The score ranges from 5 to 0, with a score of 5 indicating that the movement on the affected side is as smooth as that on the unaffected side, a score of 3 indicates that the task is possible, and a score of 0 indicates a complete lack of voluntary movement [8, 9]. A score of 1 in the SIAS Finger-Function test is further subdivided into 1a (minimal voluntary movement or mass flexion), 1b (mass extension), and 1c (minimal individual movement).

### 2.6. Statistical Analysis

One-way analysis of variance (ANOVA) was used to compare the age and days after stroke onset of each group. Chi-square tests were used to compare the sex, paralysis side, lesion type, and MAS of the biceps brachii muscle and wrist flexors.

Wilcoxon signed-rank tests were used to compare the SIAS Knee-Mouth and Finger-Function tests, FMA shoulder/elbow item, FMA wrist item, FMA finger item, upper limb total FMA score, and FIM before and after training in each group. Chi-square tests were also used to compare the MAS of the biceps brachii muscle and wrist flexors before and after training in each group, respectively.

The SIAS Knee-Mouth and Finger-Function test gains, FMA shoulder/elbow item gains, FMA wrist item, FMA finger item, and upper limb total FMA score in each group were compared among groups using the Steel–Dwass method after applying the Kruskal–Wallis test. As described previously, SIAS Finger-Function scores of 1a, 1b, and 1c transformed to 1, 2, and 3, while 2, 3, 4, and 5 in the SIAS Finger-Function score were transformed further to 4, 5, 6, and 7 to numerically treat the scores [11]. JMP® 13 (SAS Institute Inc., Cary, NC, USA) for Macintosh was used to perform the statistical analyses.

## 3. Results

A total of 101 patients were enrolled during the study period. Two patients dropped out; thus, the final analysis included 99 patients (Figure 1). We observed no significant differences in demographic data on admission among groups. The basic information of each group is shown in Table 1. The FIM motor subscore on admission was significantly higher in the NMES group compared to that in the CT group (*p* < 0.05).

The comparisons before and after training are shown in Table 2 and Figures 2 and 3. We observed no significant differences among groups in gains of SIAS Knee-Mouth test and SIAS Finger-Function test. However, the gains in FMA wrist and finger items were 0.5 and 2.0, respectively, in the RFE under NMES group, which were significantly higher than those in the CT group (*p* < 0.05). In addition, the FMA total gains also differed significantly between the RFE under the NMES and CT groups (9.0 vs. 1.0) (*p* < 0.05).

## 4. Discussion

In this study, we allocated patients with severe paretic upper limb into four groups and examined the treatment effects of NMES and/or RFE on paralysis. RFE under NMES, a repetitive exercise under continuous electrical stimulation, resulted in greater improvement in motor paralysis.

RFE uses stretch and skin-muscle reflexes to elevate the level of excitation of the injured descending motor tracts which repeated exercise rebuilds or strengthens the neural pathway reconstruction [1]. Previous studies reported that patients with moderate to mild paralysis had a significant improvement in motor paralysis in the RFE group compared to control group [1, 2]. In addition, Shimozono et al. reported that combined RFE with NMES in patients with severe paralysis significantly improved motor paralysis compared to the control group [7]. Previous report showed that FMA total gain was not significantly different between RFE with NMES and RFE; it was higher in RFE than in the control group. The results of this study were similar to the previous study; the median FMA total gain was 9 points in the RFE with NMES group, 6 points in the RFE group, 5 points in the NMES group, and 2 points in the CT group, respectively. Moreover, the RFE with NMES group improved the most; the RFE group had a higher value than the CT group. The improvement in FMA of the NMES with RFE group in the present study was 9 points and that in the Shimodozono paper was 15 points. The difference in FMA gain between the present study and previous study might be influenced by the degree of paralysis at the start of the study. It has been reported that the severity of motor paralysis in the early poststroke has a strong influence as a predictor of paralysis recovery [12, 13]. The median total FMA upper limb total score at the start of this study was 4 points, which was more severe than the 6-13 points shown in the reported by Shimodozono et al. [7] which may have affected the degree of improvement.

Besides, in previous study was a comparison between NMES under RFE, RFE, and the control group, the effect of the comparison between groups with the addition of NMES only was not clarified [7]. NMES promotes afferent inputs from the muscles to the cerebral cortex and increases the corticospinal tract excitability [14, 15]. Sugawara et al. reported enhanced motor cortex excitability when electrical stimulation was combined with voluntary movement [16]. In addition, electrically mediated repetitive movement facilitates motor relearning to make use of central neural plasticity [15]. On the other hand, it has been reported that the excitability of the cerebral cortex increases by intended muscle contractions [17]. In our study, it is speculated that RFE with NMES enhanced the excitability of the cerebral cortex by intended repetitive exercise, resulting in further improvement in motor paralysis. In particular, patients with severe paralysis with weak voluntary contraction, it is necessary to enhance the excitability of the cerebral cortex by using various techniques in order to improve the motor function. Peripheral electrical stimulation with submotor threshold stimulation intensity has been reported to improve upper limb function in stroke patients [18, 19]. In other words, when targeting patients with severe paralysis, it was considered that a method of repeated exercise while applying electrical stimulation of submotor threshold is effective for improving paralysis.

Similar to the previous study [7], the results of this study were effective in improving paralysis in the RFE under NMES group. However, there was a difference in the severity of motor paralysis between this study and previous study. The median FMA upper item scores at the start of the previous and this study were 13 and 4 points, respectively. In addition, the median gains of the total FMA points before and after the intervention were 15 points in the previous study and 9 points in this study, respectively. In previous study, each training method was matched to 40 minutes/day, performed 5 times a week for 4 weeks, the 30 minutes/day of dexterity-related training was added after each training method for all patients. Therefore, the total upper limb intervention time was 1400 minutes (70 minutes/day, 5 times a week, 4 weeks) in the previous study, the 560 minutes (20 minutes/day, 7 times a week, 4 weeks) in this study; the total amount of time was less than in previous study. Previous studies reported that there was a correlation between training time for the upper limbs and the degree of improvement of paralysis [20–22]. The difference in FMA gain between this study and the previous study is considered to be influenced by the total intervention time in addition to the severity of motor paralysis.

In our study, the RFE under the NMES group significantly improved distal motor paralysis compared to the CT group. Cui et al. reported that 12 hours a day of NMES was effective in improving wrist and finger paralysis in the paralyzed upper limb with subacute stroke patients [23]. Moreover, Lin and Yan reported that 30 minutes/day of rehabilitation focusing on the movement induced by NMES for severe paralyzed patients improved upper limb function [24]. Previous reports have reported that intervention of only electrical stimulation therapy improves the paralysis. However, their studies have performed NMES longer than this study. On the other hand, in this study, a single-channel electrical stimulator was used to perform NMES on the agonist muscle during the RFE exercise repetition, in the previous study, used multichannel electrical stimulation to apply proximal and distal to the paralyzed upper limb. It has been reported that NMES of multichannels is effective in improving paralysis [25]; it was considered that a wide area of electrical stimulation to the paralyzed muscle is effective in improving paralysis.

On the other hand, in our study, there was no significant difference between groups in the degree of improvement in proximal paralysis. Montgomery et al. reported that the trunk and proximal upper extremity muscles are also innervated by the ipsilateral cerebral cortex [26]. The tendency toward easy recovery in the proximal area may be related to the lack of difference in the degree of improvement in motor function among the treatment groups.

Improvement in paralysis reportedly depends on the frequency of use [27]. One limitation of this study was that the number of joint movement repetitions was arbitrary, although the training period of each group was defined. Therefore, additional studies are warranted to verify the effects of treatments with a fixed number of movements.

## 5. Conclusion

In the present study, RFEs under NMES was shown to be effective for severe upper limb paralysis. Especially, the therapeutic effect on the distal parts such as wrists and fingers were high. For severe paralysis with little voluntary movement, high intensity and high frequency training by the combination of RFE and NMES proved to contribute to the improvement of motor paralysis. In the future, it is necessary to make the number of operations uniform and study the effects.

## Figures and Tables

**Figure 1:** Flow diagram of this study. NMES: neuromuscular electrical stimulation; RFE: repetitive facilitative exercise; CT: conventional training.

**Figure 2:** SIAS gain comparison of each group. SIAS: Stroke Impairment Assessment Set; NMES: neuromuscular electrical stimulation; RFE: repetitive facilitative exercise; CT: conventional training. (a) SIAS Knee-Mouth test, (b) SIAS Finger-Function test. Scatter plot (circles: individual patients) and box-and-whisker plot (minimum, quartiles, and maximum) of SIAS gain in each group; scatter plot (circles: individual patients) and box-and-whisker plot (minimum, quartiles, and maximum) of SIAS gain in each group; scatter plot (circles: individual patients) and box-and-whisker plot (minimum, quartiles, and maximum) of SIAS gain in each group, black circle: outliers over 1.5 × interquartile range. No significant differences were observed between groups.

**Figure 3:** FMA item gain comparison of each group. FMA: Fugl-Meyer Assessment; NMES: neuromuscular electrical stimulation; RFE: repetitive facilitative exercise; CT: conventional training. (a) FMA upper limb total score, (b) FMA shoulder and elbow score, (c) FMA wrist score, (d) FMA finger score. Scatter plot (circles: individual patients) and box-and-whisker plot (minimum, quartiles, and maximum) of FMA gain in each group, Black circle: outliers over 1.5 × interquartile range. Significant differences were observed in the upper limb total score, wrist, and finger FMA scores between CT and NMES under RFE (^∗^*p* < 0.05, ^∗∗^*p* < 0.01).

**Table 1:** Baseline characteristics of participants.

	NMES	RFE	NMES under RFE	CT	*p* value
Number of patients	25	22	26	26	
Age (year)	57.3 ± 14.0	60.4 ± 11.5	64.1 ± 10.9	63.2 ± 13.0	n.s.
Sex (male/female)	16/9	15/7	19/7	17/9	n.s.
Paralysis side (right/left)	11/14	12/10	13/13	12/14	n.s.
Days after stroke onset	29.6 ± 12.1	31.3 ± 13.6	29.8 ± 11.6	29.4 ± 9.3	n.s.
Lesion type (ischemic/hemorrhagic)	13/12	10/12	11/15	13/13	n.s.
MAS biceps brachii (0/1/1+/2/3)	11/12/1/1/0	10/7/3/2/0	12/8/3/3/0	14/8/3/1/0	n.s.
Wrist flexors (0/1/1+/2/3)	12/10/3/0/0	10/9/2/1/0	9/13/3/1/0	10/11/4/1/0	n.s.
SIAS Knee-Mouth test	1.0 [0.0-1.0]	1.0 [0.3-2.0]	1.0 [0.0-1.0]	1.0 [0.0-1.0]	n.s.
Finger-Function test	0.0 [0.0-0.0]	0.0 [0.0-1.0]	0.0 [0.0-1.0]	0.0 [0.0-0.0]	n.s.
FMA upper limb total score	4.0 [4.0-9.0]	4.0 [4.0-8.8]	4.0 [3.0-8.8]	4.0 [4.0-5.8]	n.s.
Shoulder/elbow	0.0 [0.0-4.0]	0.5 [0.0-5.0]	0.0 [0.0-0.8]	0.0 [0.0-2.0]	n.s.
Wrist	0.0 [0.0-0.0]	0.0 [0.0-0.0]	0.0 [0.0-0.0]	0.0 [0.0-0.0]	n.s.
Finger	0.0 [0.0-0.0]	0.0 [0.0-0.0]	0.0 [0.0-0.0]	0.0 [0.0-0.0]	n.s.
FIM motor	53.0 [40.0-56.0]^∗^	47.0 [41.0-54.0]	37.5 [28.5-50.0]	35.5 [28.0-46.0]	0.02
Cognitive	27.0 [23.0-30.0]	29.0 [19.3-32.8]	24.0 [19.0-31.0]	24.5 [21.3-27.8]	n.s.
Total	76.0 [64.0-90.0]	75.0 [65.3-83.3]	64.5 [51.3-73.8]	58.0 [51.0-72.0]	n.s.

NMES: neuromuscular electrical stimulation; RFE: repetitive facilitative exercise; CT: conventional training; MAS: Modified Ashworth Scale; SIAS: Stroke Impairment Assessment Set; FMA: Fugl-Meyer Assessment; FIM: Functional Independence Measure. Continuous data are presented as mean ± SD. SIAS, FMA, and FIM scores are presented as median [lower and upper quartile]. n.s.: not significant; ^∗^significant differences in FIM motor subscore between CT and NMES (*p* < 0.05).

**Table 2:** Clinical results.

	NMES		RFE		NMES under RFE		CT	
	Pre	Post	Pre	Post	Pre	Post	Pre	Post
MAS biceps brachii (0/1/1+/2/3)	11/12/1/1	7/11/6/1	10/7/3/2	2/11/6/3^∗^	12/8/3/3	5/9/9/3	14/8/3/1	10/11/4/1
Wrist flexors (0/1/1+/2/3)	12/10/3/0	5/13/6/1	10/9/2/1	4/11/5/2	9/13/3/1	1/10/10/5^∗∗^	10/11/4/1	6/9/9/2
SIAS knee-mouth test	1.0 [0.0-1.0]	1.0 [1.0-2.0]^∗∗^	1.0 [0.3-2.0]	2.0 [1.0-2.0]^∗∗^	1.0 [0.0-1.0]	2.0 [1.0-2.0]^∗∗^	1.0 [0.0-1.0]	1.0 [0.0-2.0]^∗^
Finger-Function test	0.0 [0.0-0.0]	1.0 [0.0-1.0]^∗∗^	0.0 [0.0-1.0]	1.0 [0.0-2.0]^∗∗^	0.0 [0.0-1.0]	1.0 [0.3-2.0]^∗∗^	0.0 [0.0-0.0]	0.0 [0.0-1.0]^∗^
FMA upper limb total score	4.0 [4.0-9.0]	9.0 [5.0-18.0]^∗∗^	4.0 [4.0-8.8]	10.0 [8.3-18.8]^∗∗^	4.0 [3.0-8.8]	13.0 [9.3-22.0]^∗∗^	4.0 [4.0-5.8]	6.0 [4.0-10.8]^∗∗^
Shoulder/elbow	0.0 [0.0-4.0]	4.0 [0.0-12.0]^∗∗^	0.5 [0.0-5.0]	5.0 [4.0-11.8]^∗∗^	0.0 [0.0-0.8]	4.0 [1.3-9.5]^∗∗^	0.0 [0.0-2.0]	2.5 [0.0-6.0]^∗∗^
Wrist	0.0 [0.0-0.0]	0.0 [0.0-0.0]	0.0 [0.0-0.0]	0.0 [0.0-0.0]^∗^	0.0 [0.0-0.0]	0.5 [0.0-1.8]^∗∗^	0.0 [0.0-0.0]	0.0 [0.0-0.0]
Finger	0.0 [0.0-0.0]	1.0 [0.0-2.0]^∗∗^	0.0 [0.0-0.0]	1.0 [0.0-3.0]^∗∗^	0.0 [0.0-0.0]	2.0 [0.3-6.5]^∗∗^	0.0 [0.0-0.0]	0.0 [0.0-0.8]^∗^
FIM motor	53.0 [40.0-56.0]	69.0 [60.0-76.0]^∗∗^	47.0 [41.0-54.0]	65.0 [52.5-72.8]^∗∗^	37.5 [28.5-50.0]	52.0 [43.3-73.0]^∗∗^	35.5 [28.0-46.0]	57.5 [45.0-67.5]^∗∗^
Cognitive	27.0 [23.0-30.0]	29.0 [25.0-34.0]^∗∗^	29.0 [19.3-32.8]	29.0 [23.5-32.8]^∗∗^	24.0 [19.0-31.0]	28.0 [22.5-32.5]^∗∗^	24.5 [21.3-27.8]	25.5 [22.3-30.5]^∗∗^
Total	76.0 [64.0-90.0]	99.0 [84.0-109.0]^∗∗^	75.0 [65.3-83.3]	93.0 [81.8-101.8]^∗∗^	64.5 [51.3-73.8]	79.5 [68.0-104.3]^∗∗^	58.0 [51.0-72.0]	81.5 [70.0-98.0]^∗∗^

NMES: neuromuscular electrical stimulation; RFE: repetitive facilitative exercise; CT: conventional training; MAS: Modified Ashworth Scale; FMA: Fugl-Meyer Assessment; FIM: Functional Independence Measure. All data are presented as median [lower and upper quartile]. ^∗^Significant improvement after 4 weeks of training (^∗∗^*p* < 0.01, ^∗^*p* < 0.05).

## Data Availability

The data used to support the findings of this study are restricted by the Ethics Committee (Fujita Health University Nanakuri sanatorium Certified Review Board) in order to protect participants' privacy.
